# *Meloidogyne enterolobii* risk to agriculture, its present status and future prospective for management

This article has been retracted.

**DOI:** 10.3389/fpls.2022.1093657

**Published:** 2023-01-24

**Authors:** Aatika Sikandar, Luming Jia, Haiyan Wu, Shanshan Yang

**Affiliations:** Guangxi Key Laboratory of Agro-Environment and Agric-Products safety, College of Agriculture, Guangxi University, Nanning, China

**Keywords:** RKN, virulent, resistant, root galls, integrated disease management

## Abstract

*Meloidogyne enterolobii*, commonly known as guava root-knot nematode, poses risk due to its widespread distribution and extensive host range. This species is recognized as the most virulent root-knot nematode (RKN) species because it can emerge and breed in plants that have resistance to other tropical RKNs. They cause chlorosis, stunting, and yield reductions in host plants by producing many root galls. It is extremely challenging for farmers to diagnose due to the symptoms’ resemblance to nutritional inadequacies. This pathogen has recently been considered a significant worldwide threat to agricultural production. It is particularly challenging to diagnose a *M. enterolobii* due to the similarities between this species and other RKN species. Identified using traditional morphological and molecular techniques, which is a crucial first in integrated management. Chemical control, biological control, the adoption of resistant cultivars, and cultural control have all been developed and effectively utilized to combat root-knot nematodes in the past. The object of this study was to get about the geographical distribution, host plants, symptoms, identification, and control techniques of *M. enterolobii* and recommend future initiatives to progress its management.

## Introduction

Nematodes are one of the most abundant organisms on the planet (Hoogen et al., 2019; Sikandar et al., 2021a) and is a major component of soil (Hailu and Hailu, 2020). Plant-parasitic nematodes (PPNs) pose a significant threat to agriculture, causing an estimated yearly output loss of more than $157 billion globally (Youssef et al., 2013). The root-knot nematodes (RKN), are considered one of the most pathogenic PPN (Sikandar et al., 2019). These parasites are economically significant and one of the most destructive pests of vegetables and other crops (Tileubayeva et al., 2021). Root-knot nematodes are obligate endoparasites that live in the roots of more than 3,000 different plant species (Sikandar et al., 2020a). They are found worldwide, and their population multiplies when conditions are favorable (Feyisa, 2022).

*Meloidogyne enterolobii*, known as guava root-knot nematode, poses a risk to agriculture because of its worldwide distribution and diverse host range (Dareus et al., 2021). This species is recognized as being among the most virulent RKNspecies due to its ability to emerge and breed in host plants having resistance against major tropical RKN (Koutsovoulos et al., 2020). *M. enterolobii* was previously identified as *M. incognita* in 1983 in the Chinese pacara earpod tree (*Enterolobium contortisiliquum*) (Yang and Eisenback, 1983). In 1988, it was represented as a novel species found in Puerto Rico, identified as *Meloidogyne mayaguensis* (Rammah and Hirschmann, 1988). However, in 2004 it was reclassified as *Meloidogyne enterolobii* based on morphological and molecular evidence (Xu et al., 2004). This nematode had caused tremendous harm in the *Psidium guajava* (guava trees) in South America, that’s why it commonly called “guava root-knot nematode” (Palomares-Rius et al., 2021). *M. enterolobii* may cause more than 65% of the losses alone, which is significantly greater than any other RKNs species (Castagnone-Sereno, 2012). The growers still may not recognize that crops infecteduntil the harvest occurs and then notice a high number of galls on roots (Philbrick et al., 2020). Because of the similarities between *M. enterolobii* and other RKN species, diagnosing an infestation of *M. enterolobii* is very difficult (Min et al., 2012).

Synthetic chemicals have been used to control nematodes, but they are very poisonous and hazardous to the environment (Sikandar et al., 2021b). Most nematicide compounds, including ethylene dibromide (EDB), dibromochloropropane, and methyl bromide have been withdrawn from the market because several are carcinogenic (Onkendi et al., 2014). Bio-control, crop rotation, cultural practices, and plant resistance are now the main research areas for researchers attempting to address this challenging problem (Sikandar et al., 2020b). Compared to chemicals, bio-control is safer and more environmentally friendly because it has no residual effect (Köhl et al., 2019).

Thus, we present an overview of *M. enterolobii* research from all over the world. Moreover, we focused on how this accomplishment can help with *M. enterolobii* control. This review also includes species details as well as some recommendations for additional research on this lethal pathogen.

## Geographical distribution and host plants

*Meloidogyne enterolobii* nematode has been documented globally and is primarily found in tropical and subtropical areas (Silva and Santos, 2017). However, it was discovered in China and has now been recorded in Africa, Asia, Amercia (North and South) and Europe (**Table 1**).

**Table 1:** Geographic distribution of *Meloidogyne enterolobii*.

Continent	Country	Reference
Africa	Cote d’Ivoire	Fargette (1987)
	Togo	Fargette (1987)
	Burkina Faso	Fargette et al. (1994)
	Senegal	Diop (1994)
	South Africa	Willers (1997)
	Malawi	Trudgill et al. (2000)
	Congo	Onkendi et al. (2014)
	Nigeria	Kolombia et al. (2016)
	Kenya	Chitambo et al. (2016)
	Niger	Assoumana et al. (2017)
	Benin	Affokpon et al. (2017)
	Mozambique	Kisitu et al. (2017)
America (North)	Guadeloupe	Rammah and Hirschmann (1988)
	Puerto Rico	Rammah and Hirschmann (1988)
	Cuba	Decker and Rodriguez Fuentes (1989)
	Guatemala	Carneiro et al. (2000)
	Martinique	Carneiro et al. (2000)
	United State of America	Brito et al. (2004)
	Costa Rica	Humphreys et al. (2012)
America (South)	Trinidad and Tobago	Trudgill et al. (2000)
	Brazil	Carneiro et al. (2001)
	Venezuela	Lugo et al. (2005)
Asia	China	Yang and Eisenback (1983)
	Vietnam	Iwahori et al. (2009)
	Thailand	Jindapunnapat (2012)
	India	Poornima et al. (2016)
Europe	Switzerland	Kiewnick et al. (2008)
	Portugal	Santos et al. (2019)

It is a polyphagous RKN with various plant host species (**Table 2**). Only a few number of fruit and vegetable species (*Allium fistulosum, A. sativum, Anacardium occidentale, Annona cherimola, Arachis hypogaea, Averrhoa carambola, Brassica oleracea, Citrus aurantium, Citrus limonia, Citrus paradise, Citrus reticulate*, *C. reticulate, C. sunki, C. trifoliate*, *C. volkameriana, Cocos nucifera, Euterpe oleracea, Fragaria ananassa, Mangifera indica, Olea europaea, Passiflora* spp.*, Persea americana and Zea mays*) have been documented to be poor hosts for *M. enterolobii* (Freitas et al., 2017; EPPO-Datasheet, 2020).

**Table 2:** *Meloidogyne enterolobii* host plants reported worldwide.

Scientific name	Common name	Family	References
*Abelmoschus esculentus*	Okra	Malvaceae	Vinícius-Marin et al. (2017)
*Acalypha australis*	Copperleaf	Euphorbiaceae	Jia et al. (2022)
*Acanthospermum australe*	Spiny-bur	Asteraceae	Bellé et al. (2019)
*Ajuga reptans*	Bugleweed	Lamiaceae	Brito et al. (2010)
*Allium porrum*	Garden leek	Amaryllidaceae	Rosa et al. (2015)
*Amaranthus deflexus*	Perennial pigweed	Amaranthaceae	Bellé et al. (2019)
*A. hybridus*	Pigweed		Rich et al. (2009)
*A. spinosus*	Spiny amaranth		Rich et al. (2009)
*A. tricolor*	Edible amaranth		Bellé et al. (2019)
*Ananas comosus*	Pineapple	Bromeliaceae	Silva and Oliveira (2010)
*Angelonia angustifolia*	Summer Snapdragon	Plantaginaceae	Kaur et al. (2006)
*Apium graveolens*	Celery	Apiaceae	Rodriguez et al. (2003)
*Artocarpus heterophyllus*	Jackfruit	Moraceae	Brito et al. (2015)
*Beta vulgaris*	Sugar beet	Chenopodiaceae	Moens et al. (2009)
*Bidens pilosa*	Hairy beggar ticks	Asteraceae	Bellé et al. (2019)
*Brassica oleracea*	Mustard	Brassicaceae	Bitencourt and Silva (2010)
*Brugmansia suaveolens*	White angel trumpet	Solanaceae	Brito et al. (2010)
*Buddleja davidii*	Butterfly bush	Scrophulariaceae	Brito et al. (2010)
*Byrsonima cydoniifolia*	Nanche	Malpighiaceae	Paes et al. (2012)
*Cactus* sp.	Cactus	Cactaceae	Silva et al. (2016)
*Callistemon citrinus*	Lemon bottlebrush	Myrtaceae	Brito et al. (2010)
*C. rigidus*	Stiff bottlebrush		Marques et al. (2012)
*C. viminalis*	Weeping bottlebrush		Brito et al. (2010)
*Cannabis sativa*	Hemp	Cannabaceae	Ren et al. (2021)
*Canavalia ensiformis*	Jack bean	Fabaceae	Moens et al. (2009)
*Capsicum annuum*	Bell pepper	Solanaceae	Assoumana et al. (2017)
*Capsicum baccatum*	Orchid pepper	Solanaceae	Pinheiro et al. (2014)
*Capsicum chinense*	Habanero pepper	Solanaceae	Melo et al. (2011)
*Capsicum frutescens*	Bird pepper	Solanaceae	Silva et al. (2016)
*Carica papaya*	Papaya	Caricaceae	Freitas et al. (2017)
*Caryopteris clandonensis*	Bluebeard	Lamiaceae	Brito et al. (2010)
*Cassia occidentalis*	Coffee Senna	Caesalpiniacea	Mendes and Dickson (2016)
*Cereus fernambucensis*	Cactus	Cactaceae	Souza et al. (2006)
*Chamaesyce hypericifolia*	Graceful spurge	Euphorbiaceae	Quénéhervé et al. (2011)
*Citrullus lanatus*	Watermelon	Cucurbitaceae	Ramírez-Suárez et al. (2014)
*Coffea arabica*	Coffee	Rubiaceae	Muniz et al. (2008)
*Commelina benghalensis*	Wandering Jew	Commelinaceae	Bellé et al. (2019)
*Coriandrum sativum*	Coriander	Apiaceae	Bitencourt and Silva (2010)
*Cucumis melo*	Sweet melon	Cucurbitaceae	Freitas et al. (2017)
*C. sativus*	Cucumber		Bitencourt and Silva (2010)
*Cucurbita moschata*	Pumpkin	Cucurbitaceae	Marques et al. (2012)
*Daucus carota*	Carrot	Apiaceae	Wang et al. (2014)
*Dioscorea rotundata*	Yam	Dioscoreaceae	Kolombia et al. (2016)
*Elaeocarpus decipiens*	Japanese blueberry	Elaeocarpaceae	Moore et al. (2020)
*Emilia sonchifolia*	Lilac Tassel Flower	Asteraceae	Rich et al. (2009)
*Enterolobium contortisiliquum*	Tamboril	Fabaceae	Yang and Eisenback (1983)
*Erechtites hieraciifolius*	American burnweed	Asteraceae	Carneiro et al. (2006)
*Euphorbia heterophylla*	Desert spurge	Euphorbiaceae	Silva and Krasuski (2012)
*E. prostrata*	Ground spurge		Rich et al. (2009)
*E. punicea*	Jamaican poinsettia		Han et al. (2012)
*E. tirucalli*	Indian tree spurge		Souza et al. (2006)
*Fatoua villosa*	Mulberryweed	Moraceae	Brito et al. (2008)
*Ficus carica*	Common fig	Moraceae	Freitas et al. (2014)
*Galinsoga parviflora*	Potato weed	Asteraceae	Bellé et al. (2019)
*Gardenia jasminoides*	Cape jasmine	Rubiaceae	Lu et al. (2019)
*Glycine max*	Soybean	Fabaceae	Ye et al. (2013)
*Gossypium hirsutum*	Cotton	Malvaceae	Ye et al. (2013)
*Helianthus* sp.	Sunflower	Asteraceae	Rosa et al. (2015)
*Hibiscus grandiflorus*	Swamp rose mallow	Malvaceae	Brito et al. (2010)
*Hydrocotyle bonariensis*	Largeleaf pennywort	Araliaceae	Souza et al. (2006)
*Hypericum* sp.	St. John’s wort	Hypericaceae	Silva et al. (2016)
*Inga edulis*	Ice-cream bean	Fabaceae	Silva et al. (2016)
*Ipomoea batatas*	Sweet potato	Convolvulaceae	Melo et al. (2011)
*Ixora chinensis*	Chinese Ixora	Rubiaceae	Wu et al. (2022a)
*Jatropha urens*	Bull nettle	Euphorbiaceae	EPPO-Datasheet (2020)
*Lactuca sativa*	Garden lettuce	Asteraceae	Correia et al. (2015)
*Lagerstroemia indica*	Crape myrtle	Lythraceae	Brito et al. (2010)
*Lampranthus* sp.	Ice plant	Aizoaceae	EPPO-Datasheet (2020)
*Lantana camara*	Shrub lantana	Verbenaceae	Silva et al. (2016)
*L. montevidensis*	Weeping lantana		Brito et al. (2010)
*Leonotis nepetifolia*	Christmas candlestick	Lamiaceae	Quénéhervé et al. (2011)
*Leonurus sibiricus*	Siberian motherwort	Lamiaceae	Bellé et al. (2019)
*Ligustrum* sp.	Privet	Oleaceae	Brito et al. (2010)
*Luffa cylindrica*	Sponge gourd	Cucurbitaceae	Marques et al. (2012)
*Lycopersicon peruvianum*	Peruvian tomato	Solanaceae	Melo et al. (2011)
*L. hirsutum*	Hairy tomato		Melo et al. (2011)
*Malpighia emarginata*	Acerola cherry	Malpighiaceae	(Humphreys et al., 2012)
*M. glabra*	Barbados cherry		Silva et al. (2016)
*Manihot esculenta*	Cassava	Euphorbiaceae	Rosa et al. (2014)
*Maranta arundinacea*	Arrow root	Marantaceae	Zhuo et al. (2010)
*Melaleuca linearis*	Pine-leave bottlebrush	Myrtaceae	EPPO-Datasheet (2020)
*M. viminalis*	Weeping Bottlebrush		EPPO-Datasheet (2020)
*Merremia aegyptia*	Hairy woodrose	Convolvulaceae	Cunha e Castro (2019)
*Mesona chinensis*	Chinese mesona	Lamiaceae	Wu et al. (2022a)
*Morinda citrifolia*	Indian mulberry	Rubiaceae	Brito et al. (2010)
*Morus alba*	White mulberry	Moraceae	Sun et al. (2019)
*M. celtidifolia*	Texas mulberry		Soares et al. (2018)
*M. nigra*	Black mulberry		Paes-Takahashi et al. (2015)
*Musa* spp.	Banana	Musaceae	Freitas et al. (2014)
*Myrica cerifera*	Wax myrtle	Myricaceae	Brito et al. (2010)
*Nicandra physaloides*	Apple of Peru	Solanaceae	Bellé et al. (2019)
*Nicotiana tabacum*	Tobacco	Solanaceae	Moens et al. (2009)
*Ocimum basilicum*	Thai basil	Lamiaceae	Gu et al. (2021)
*Oeceoclades maculata*	Monk orchid	Orchidaceae	Carneiro et al. (2006)
*Ormosia hosiei*	Horse-eye bean	Fabaceae	Wu et al. (2022b)
*Panicum* sp.	Panic Grass	Poaceae	Brito et al. (2008)
*Passiflora mucronata*	Passion Flower	Passifloraceae	Rich et al. (2009)
*Paulownia elongata*	Empress tree	Paulowniaceae	EPPO-Datasheet (2020)
*Pentas lanceolata*	Star Cluster	Rubiaceae	Brito et al. (2010)
*Phaseolus vulgaris*	Common bean	Fabaceae	Moens et al. (2009)
*Physalis angulata*	Cutleaf ground cherry	Solanaceae	Marques et al. (2012)
*P. peruviana*	Cape gooseberry		Castagnone-Sereno (2012)
*Psidium guajava*	Guava	Myrtaceae	Almeida et al. (2010)
*P. guineense*	Brazilian guava		Marques et al. (2012)
*P. myrtoides*	Guava		Marques et al. (2012)
*Punica granatum*	Pomegranate	Punicaceae	Silva and Krasuski (2012)
*Raphanus sativus*	Radish	Brassicaceae	Rosa et al. (2014)
*Rhynchelytrum repens*	Natal grass	Poaceae	Bellé et al. (2019)
*Rosa* sp.	Rose	Rosaceae	EPPO-Datasheet (2020)
*Rotheca myricoides*	Butterfly bush	Lamiaceae	EPPO-Datasheet (2020)
*Saccharum* sp.	Sugarcane	Poaceae	Marques et al. (2012)
*Salix* sp.	Willow	Salicaceae	Brito et al. (2010)
*Salvia leucantha*	Mexican bush sage	Lamiaceae	Levin et al. (2005)
*Senna alata*	Candle bush	Fabaceae	Souza et al. (2006)
*S. occidentalis*	Coffee senna		Souza et al. (2006)
*Sida rhombifolia*	Arrow leaf sida	Malvaceae	Bellé et al. (2019)
*Solandra maxima*	Hawaiian lily	Solanaceae	Brito et al. (2010)
*Solanum americanum*	American black nightshade	Solanaceae	Pinheiro et al. (2019)
*S. gilo*	Scarlet eggplant		Marques et al. (2012)
*S. lycopersicum*	Tomato		Silva et al. (2020)
*S. melongena*	Aubergine		Ghule et al. (2020)
*S. pseudocapsicum*	Jerusalem cherry		Groth et al. (2017)
*S. quitoense*	Naranjilla		Ghule et al. (2020)
*S. scabrum*	Garden huckleberry		EPPO-Datasheet (2020)
*S. sisymbriifolium*	Sticky nightshade		Bellé et al. (2019)
*S. paniculatum*	Jurubeba		Silva and Santos (2017)
*S. pseudocapsicum*	Jerusalem cherry		Groth et al. (2017)
*S. tuberosum*	Potato		Kan et al. (2008)
*Stenocereus queretaroensis*	Pitaya	Cactaceae	Ramírez-Suárez et al. (2016)
*Syngonium* sp.	Arrowhead plant	Araceae	EPPO-Datasheet (2020)
*Syzygium aromaticum*	Clove	Myrtaceae	EPPO-Datasheet (2020)
*Talinum patens*	Jewels of Opar	Talinaceae	Groth et al. (2017)
*T. fruticosum*	Ceylon spinach		EPPO-Datasheet (2020)
*T. triangulare*	Philippine spinach		Souza et al. (2006)
*Tecoma capensis*	Cape honeysuckle	Bignoniaceae	Moens et al. (2009)
*Tibouchina elegans*	Glory bush	Melastomataceae	Moens et al. (2009)
*Ulmus parvifolia*	Chinese elm	Ulmaceae	Quénéhervé et al. (2011)
*Washingtonia* sp.	Washington fanpalm	Arecaceae	Brito et al. (2010)
*Vigna unguiculata*	Cowpea	Fabaceae	Guimarães et al. (2003)
*Zingiber officinale*	Ginger	Zingiberaceae	Xiao et al. (2018)
*Zizyphus jujuba*	Chinese date	Rhamnaceae	Long et al. (2014)

## Symptoms

Plants infected with *M. enterolobii* have reduced growth, life span, and resistance against several abiotic stresses (Dareus et al., 2021). Generally, *M. enterolobii* effects may include reduced yield quality and quantity (Abd-Elgawad, 2021). Above-ground symptoms include leaf yellowing, wilting, and stunted growth while below-ground symptoms, such as root galls, can be considerable in size and quantity (Jia et al., 2022). Plants infected by *M. enterolobii* are more vulnerable to secondary plant infections, such as *Fusarium solani* parasitizing guava after infestation (Gomes et al., 2014).

## Identification of *Meloidogyne enterolobii*

### Morphology

Species of *Meloidogyne* have been identified based on adults’ morphology, along with an examination of the perineal patterns, which are structures of cuticle folds around the anus and vulva in adult females (Archidona-Yuste et al., 2018). Such detection techniques need tremendous experience and expertise, and negligence in using them may result in misdiagnosis (Bogale et al., 2020). The perineal patterns’ characteristics effectively distinguish *M. enterolobii* from other species of *Meloidogyne* (Ydinli and Mennan, 2016). *M. enterolobii* perineal patterns are often oval, with a round and high dorsal arch, large phasmids, a round tail tip part that lacks striae, and sometimes weak lateral lines present (Hunt and Handoo, 2009). Furthermore, perineal patterns within the species might differ between individuals, making diagnosis difficult (Karssen and Van Aelst, 2001). Moreover, *M. enterolobii* and *M. incognita* can exhibit eerily alike perineal patterns (Iwahori et al., 2009; Cunha et al., 2018), which is why *M. enterolobii* was initially believed to be *M. incognita* based upon the perineal investigation. Female RKN may be distinguished by their stylet, neck length, body form, and perineal pattern (Subbotin et al., 2021). Body morphometrics can be used to identify males and second-stage juveniles (J2) (Nyaku et al., 2018). Most RKN species have overlapping characteristics and measurements, making species identification challenging (Maleita et al., 2018).

### Isozyme analysis

Isozyme analysis is a biochemically standard diagnostic procedure that involves staining and observing malate dehydrogenase (Mdh), esterase, and cellulose acetate isozyme profiles after separation and migration through the electrophoresis (Siddiquee et al., 2010). The inter-species diversity produces a lot of isozymes, which have the same catalytic roles but differing chemical characteristics, like mobility in electrophoresis (Simonsen, 2012). The distinct pattern of one Mdh band and two distinct esterase bands in *M. enterolobii* distinguishes it from other species (Palomares-Rius et al., 2021). This approach successfully differentiated young adult females into species, while not being applicable for J2s (Castillo and Castagnone-Sereno, 2020). Additionally, this is extremely sensitive and carried out using only one adult female’s isolated protein (Birithia et al., 2012). Even though isozyme investigation was commonly used for identification of *Meloidogyne* (Nisa et al., 2022), more than single polymorphic enzyme was required to authenticate the identification of specific isolates because the presence or absence of an enzyme signal could varywithin and between samples (Cunha et al., 2018).

### Species specific polymerase chain reaction assay

This method has been designed and employed to distinguish the RKN species (Bhat et al., 2022). *M. enterolobii* was identified using a sequence characterized amplified region (SCAR) primer pair, such as MK7F/MK7R (GATCAGAGGCGGGCGCATTGCGA/CGAACTCGCTCGAACTCGAC) (Tigano et al., 2010). The IGS2 primers MeF/MeR (AACTTTTGTGAAAGTGCCGCTG/TCAGTTCAGGCAGGATCAACC) were substantially specific than MK7F/MK7R primers (Villar-Luna et al., 2016). TW81F/AB28R internal transcribed spacer (ITS) region primers were employed to diagnose *M. enterolobii* (Suresh et al., 2019). The multiplex PCR was intended to diagnose *M. javanica*, *M. enterolobii*, and *M. incognita* by DNA obtained directly from a single gall at different life cycle stages (Hu et al., 2011). A quantitative real-time PCR (qPCR) technique that measures the quantity of nucleic acid presence was developed for the precise detection, identification, and possibly quantification of *M. enterolobii* in both host roots and soil (Sapkota et al., 2016). In *M. enterolobii*, a unique satellite DNA family called pMmPet was found, providing species-specific PCR, dot blot, and southern blot analysis identification (Braun-Kiewnick et al., 2016). It was discovered that the satellite repetition was highly abundant and persistent across various populations of *M. enterolobii*, enabling single-individual identification and rendering it an efficient screening tool (Philbrick et al., 2020).

### Loop-mediated isothermal amplification

This approach has been designed to amplify DNA with selectivity, sensibility, accuracy, and quickly in isothermal conditions (Cai et al., 2018). Moreover, LAMP could amplify DNA in 1 hour in isothermal conditions using two or three sets of primers (Chen et al., 2011). A simple screening technique designed and employed in the field to detect *M. enterolobii*, *M. arenaria*, *M. hapla*, *M. javanica*, and *M. incognita* is recognized as the LAMP assay (Niu et al., 2012). Using a single-tube assay method based on the PCR melting curve methodology, the novel post-PCR analysis approach known as high-resolution melting curve analysis (HRMC) may distinguish between different DNA sequences according to their length, composition, and GC content (Holterman et al., 2012). Various tropical *Meloidogyne* species might be distinguished using HRMC analysis (Palomares-Rius et al., 2021). *M. enterolobii* isolates displayed distinct melting peak trends, having 1 or 2 peaks with varying centered heights at various melting temperatures, indicating a risk of employing a fragment that generated multiple amplicons of different lengths inside the same species (Chen et al., 2022). Moreover, examining novel single copy genes and regions in multiplex HRMC tests may be efficient in distinguishing *M. enterolobii* from other RKN species (Chen et al., 2022). Single nucleotide polymorphisms (SNPs) analysis may be an effective and reasonable method for diagnosing *M. enterolobii* (Holterman et al., 2012). The phylogenetic genetic relationships of the *M. javanica*, *M. enterolobii*, and *M. incognita* populations in South Africa were successfully investigated, and 34 SNPs that effectively distinguished these *Meloidogyne* species were discovered by using the genotyping-by-sequencing (GBS) technique (Rashidifard, 2019). Koutsovoulos et al. (2020) reported the genomes of *M. hapla*, *M. incognita*, and *M. enterolobii*. Because mitotic parthenogenesis is also a mode of reproduction in *M. enterolobii*, there has been little genetic variability found inside it (Humphreys-Pereira and Elling, 2015). The *M. enterolobii* isolates from various hosts and regions were tested using DNA markers, which revealed that they were genetically homogenous (Schwarz et al., 2020).

## Life cycle

*M. enterolobii’s* life cycle (**Figure 1**)is similar to other RKN species (Castillo and Castagnone-Sereno, 2020). Mature females lay their eggs in a gelatinous matrix (Kole, 2020). This matrix holds the eggs together, which protects them from severe climatic conditions (Mwesige, 2013). The nematode develops into a first-stage juvenile (J1), then molts into J2, and then hatchs from the egg (Velloso et al., 2022). Hatching can be affected by moisture, temperature, and the pH of the soil (Velloso et al., 2022). Second-stage juveniles travel toward the new host and penetrate the root system (Rashidifard et al., 2021). These nematodes travel to the vascular cylinder, and make massive feeding sites by causing physical damage with the stylets and releasing cellulolytic and proteolytic enzymes (Pulavarty et al., 2021). Giant cells form on the feeding sites, resulting in the characteristic galls observed on infected root systems (Nguyen, 2016). Giant cells are multinucleated, larger cells that normally develop in plant vascular tissues, and nourish nematodes by redistributing the metabolites of plants (Sreekavya et al., 2019). The J2 further molt three times, transitioning to the third-stage (J3) and fourth-stage (J4) until becoming sexual adults (Jagdale et al., 2021). Due to a malfunctioning stylet, the J3 and J4 stage nematodes cannot feed (Rashidifard, 2019). Vermiform male *M. enterolobii* worms emerge from the root system of the host plant (Castillo and Castagnone-Sereno, 2020). Furthermore, various *Meloidogyne* species only develop males in non-favorable circumstances, like extremely hot soil and inadequate moisture content (Giné et al., 2021). The *Meloidogyne* species have a 30-35 days life cycle in ideal circumstances, and every female may produce 500-1000 eggs in a gelatinous matrix (Feyisa, 2022). Koutsovoulos et al. (2020) demonstrated that *M. enterolobii* can also reproduce by obligate mitotic parthenogenesis, which occurs when the nucleus splits into two daughter nuclei that share similar genetic information as their parents. Meanwhile males can arise from genetically predisposed females under harsh environmental circumstances (Philbrick et al., 2020).

**Figure 1:** Life cycle of Meloidogyne enterolobii.

## Disease incidence condition

The incidence of the disease and yield losses caused by root-knot nematodes are frequently undetermined because their foliar signs are identical to those of other biotic diseases and abiotic stresses, such as stunted growth and yellow leaves (Liang et al., 2020). *M. enterolobii* is an extremely pathogenic species that causes extensive root galling as compared to other *Meloidogyne* species. It is also a very effective parasitic species with a high infestation rate on the host plant’s roots. Tomato yield declined by up to 65% in a microplot experiment (Cetintas et al., 2008). In just two greenhouses in Switzerland, output losses of up to 50% and substantial stunting of cucumber and tomato rootstocks were observed (Kiewnick et al., 2008). Infected Mulberry (*Morus* spp.) plants developed many galls on their roots, which are characteristic indications of root-knot nematode (*M. enterolobii*) infection, and the disease incidence was 100% (Sun et al., 2019). *M. enterolobii* reduced guava production in Brazil by 70% in 7 years, resulting in a US$61 million economic loss, that’s why cultivation may become unprofitable in highly infested areas with *M. enterolobii* (Carneiro et al., 2007).

## Integrated disease management strategies

It includes the combined application of several disease management strategies in order to reduce disease prevalence and severity while also reducing the pathogenic population below the devastating economic threshold (Forghani and Hajihassani, 2020). While integrated disease management (IDM) is a cost-effective and environmentally friendly strategy, it might be difficult to control the disease when a severe *M. enterolobii* infection has developed (Schwarz et al., 2020). *M. enterolobii* management is difficult because of its diverse host range and rapid reproduction cycles (Castagnone-Sereno, 2012). Therefore, developing successful strategies and incorporating them into disease management programs might effectively prevent disease outbreaks, lower disease severity, and boost agricultural output (Desaeger et al., 2020). They can be managed using various methods, such as chemical control, biological control, the adoption of resistant cultivars, and cultural control (Abd-Elgawad, 2022). The researchers usually use a single management strategy at a time to control this virulent nematode, so there is an urgent need to design a study in which different management strategies are applied at a time and also focus on inventing new management strategies. Additionally, a reliable and accurate diagnostic technique for *M. enterolobii* investigation might promote agricultural productivity and improve preventative activities to protect epidemiological research and crop management strategies internationally.

### Chemical control

The application of chemical nematicides has controlled *Meloidogyne* species, although most of these substances are being banned due to safety concerns and hazards (Abd-Elgawad, 2021). Non-fumigants and fumigants are two major chemical nematicides used to regulate *M. enterolobii* (Castillo and Castagnone-Sereno, 2020). Non-fumigant nematicides are often prepared as liquids or grains form that can be properly mixed in water (Morris, 2015). Ethoprop, fluopyram, terbufos, fluensulfone, and oxamyl are some popular non-fumigant nematicides that are often used to manage *Meloidogyne* species (Desaeger et al., 2020). While the fumigants are typically composed of gases or liquids, this enables them to be rapidly evaporated and circulate in air holes between soil particles (Stejskal et al., 2021). The fumigants 1,3-dichloropropene, metam sodium, and metam potassium are commonly used to control *M. enterolobii* (Talavera-Rubia and Verdejo-Lucas, 2021). While fumigants are effective in controlling *Meloidogyne* species, these are generally costly and vulnerable to heightened legal scrutiny (Nyczepir and Thomas, 2009). Moreover, nematicides are classified as contact or systemic based on whether they directly kill nematodes in the soil or are first absorbed by plants (Lahm et al., 2017). Such chemical nematicides are incredibly hazardous as their residues can be detected in the food chain (Abd-Elgawad, 2016). Nematicide mode of action refers to the lethal action of nematicides on important life processes within nematode (Oka, 2020). Broad-spectrum fumigant nematicides, enter the nematode’s body wall directly and do not need to be eaten to be effective (Desaeger et al., 2020). Once they enter the nematode’s body cavity, they affect various internal organs when these organs are drenched in body fluids containing the nematicide (Desaeger et al., 2020). However, they are characterized biocidal compounds because they effect on fungus, bacteria, seeds, and other organisms in the soil and can pose environmental disruption and phyto-toxicity (Ebone et al., 2019; Oka, 2020). Nonfumigants can also directly enter nematodes’ body walls (Ebone et al., 2019).

### Biological control

Biological control with microbial antagonists (bacteria and fungi) has generated tremendous attention as a safe alternate and potential method of controlling plant-parasitic nematodes for ecological balance and safety (Riascos-Ortiz et al., 2022). *Bacillus firmus*, *B. firmus*, *B. amyloliquefaciens*, *B. subtilis*, *B. urkholderia* spp., *Microbacterium* spp., *Paenibacillus* spp., *Pseudomonas* spp., *Serratia* spp., *Sinorhizobium* spp., and *Streptomyces* spp. have exhibited nematicidal action against eggs, juveniles, and adults of *Meloidogyne* species (Aioub et al., 2022). *Paenibacillus alvei* increased the mortality of juveniles and decreased the hatching of *M. enterolobii* (Bakengesa, 2016). *Microbacterium maritypicum* and *Sinorhizobium fredii* have been shown to restrain nematode development and promote systemic resistance (Zhao et al., 2019). Plant-parasitic nematodes *M. enterolobii* are suppressed by plant growth promoting bacteria (PGPB) *via* several processes depending on microorganisms’ ability to compete successfully for ecological niches, colonize plant surfaces, and release nematicidal and antimicrobial chemicals (hydrolytic enzymes, toxins, antibiotics, siderophores, etc.) (Bakengesa, 2016; Gamalero and Glick, 2020). Bacteria and their metabolites have an impact on both the plant and microbial communities (Burkett-Cadena et al., 2008). Antibiosis, parasitism, or competition for resources or infection sites can all have a direct antagonistic effect (Migunova and Sasanelli, 2021). Bacteria can indirectly boost host defensive systems, resulting in induced systemic resistance (ISR) (Yu et al., 2022). *Acremonium*, *Arthrobotrys*, *Chaetomium*, *Monacrosporium*, *Paecilomyces*, *Pochonia*, *Purpureocillium*, and *Trichoderma* are fungi that are antagonistic and trap nematodes with sticky mycelia (Moliszewska et al., 2022). Endophytic fungi like *Paecilomyces* and *Trichoderma* can capture and destroy *Meloidogyne* species in the soil or root systems and restrain their development (Kassam et al., 2022). Similarly, *Purpureocillium lilacinum* and *Pochonia chlamydosporia* display the most significant effects and are suitable for biocontrol of *M. enterolobii* (Flores Francisco et al., 2021). To control *M. enterolobii*, additional study is required on the efficiency and broad-spectrum action, improving growth conditions, and sustainability of beneficial antagonistic bacteria or fungi for their marketing and use in IDM. Arbuscular mycorrhizal fungi (AMF) form a mutualistic symbiotic relationship with plants. As a result, they alter root structure, increasing plant tolerance, altering rhizosphere interactions, limiting plant-parasitic nematode feeding and space in the root, and inducing systemic resistance (ISR) (Vishwakarma et al., 2022). As microbiome research expands, the discovery of beneficial microbial agents for *M. enterolobii* for field application will be critical in the coming years (Galileya Medison et al., 2021). It is also crucial to consider how beneficial microbes interact with plant roots and symbiotic connections to better understand the various mechanisms behind their activities against *M. enterolobii* (Mohamed et al., 2022). According to research on its direct effects on plant-parasitic nematodes and its numerous benefits, AMF may be utilized as a biocontrol agent in suppressing *M. enterolobii* and improving nutrient absorption for improved crop productivity and quality (Forghani and Hajihassani, 2020). Fungi are recognized as a biocontrol agent through various mechanisms of action, including antibiosis, mycoparasitism, competition with pathogens, stimulation of plant growth, improved plant tolerance to abiotic stressors, and activation of pathogen defenses (Hermosa et al., 2012). The major direct contact mechanisms are competition and the formation of lytic enzymes and/or secondary metabolites (antibiosis) (Poveda, 2020). In order to colonize plant tissues, endophytic fungi must at least partially inhibit the plant defenses that allow them to produce induced systematic resistance (ISR) and systematic acquired resistance (SAR) against the invasion of pests and/or diseases (Busby et al., 2016). The strictly direct mechanisms of mycorrhizal fungi against nematodes are not yet adequately described, as they typically act through the plant host, altering root morphology by increasing root growth and branching, increasing water uptake and nutrients, making plants competitive with other plants for nutrients and space, or changing rhizosphere interactions (Schouteden et al., 2015). Nematodes can be directly attacked, killed, rendered immobile, or repelled by endophytic fungi. They can also be rendered unable to locate their hosts, have an effect on the development of nurse cells, compete in resource competition, or combine several of these tactics (Schouten, 2016).

### Resistance

Numerous research projects are being conducted worldwide to improve plant resistance to RKN (Padilla-Hurtado et al., 2022). The most cost-effective and environmentally friendly way to eradicate RKNs is to plant resistant cultivars (Ayala-Doñas et al., 2020). *Meloidogyne* species resistance is conferred by at least ten plant-resistance genes (Mi-1, Mi-2, Mi-3, Mi-4, Mi-5, Mi-6, Mi-7, Mi-8, Mi-9, and Mi-HT) (Rezk et al., 2021). Only five of them (Mi-1, Mi-3, Mi-5, Mi-9, and Mi-HT) have now had their genes mapped (El-Sappah et al., 2019). However, *M. enterolobii* is more pathogenic than other *Meloidogyne* species in crop genotypes with multiple sources of resistance genes (Collett et al., 2021). For instance, *M. enterolobii* thrives in crop genotypes resistant to other *Meloidogyne* species, such as resistant *Capsicum annuum* (N gene, Tabasco gene), *Vigna unguiculata* (Rk gene), *Glycine max* (Mir1 gene), *Gossypium hirsutum, Ipomoea batatas, Solanum lycopersicum* (Mi-1 gene), and *Solanum tuberosum* (Mh gene) (Schwarz, 2019).

Currently, researchers have concentrated on finding alternative sources of genetic resistance against *M. enterolobii* because this species has the potential to reproduce on a variety of crops that have resistance genes against other nematodes species (Castillo and Castagnone-Sereno, 2020). The exploration of new sources of tolerance or resistance against *M. enterolobii* has required a tremendous amount of research. In the previous research, Silva et al. (2019) reported that three varieties of wild and commercial tomatoes (*Solanum pimpinellifolium* “CGO 7650”, and *S. lycopersicum* “CNPH 1246 and Yoshimatsu”) exhibited resistance against *M. enterolobii*. Pinheiro et al. (2020) studied thirty-seven pepper genotypes to identify their resistance against three root-knot nematode species (*M. incognita*, *M. javanica*, and *M. enterolobii*). Only two genotypes (CNPH 6144 and CNPH 30118) were resistant against *M. enterolobii*.

Moreover, translationally controlled tumor protein (TCTP) was initially discovered in mice (Yenofsky et al., 1982). A new *M. enterolobii* TCTP (MeTCTP) effector exhibited the potential to increase parasitism, most likely by reducing programmed cell death in the host (Zhuo et al., 2017). The silencing of the MeTCTP effector reduced the reproduction and parasitic ability of *M. enterolobii*, indicating the nematode effector gene as a target for host-generated RNAi to establish disease resistance (Zhuo et al., 2017). Furthermore, new bioinformatics tools and genome sequence data have both become available for efficient dsRNA construction and stacking dsRNA sequences to target several genes for management of nematodes (Banerjee et al., 2017). The identification and functional studies of nematode-effector targets utilizing RNAi technology could carry substantial potential to enhance resistance in plants to *M. enterolobii*.

### Cultural control

Cultural control is an old and cost-effective approach to manage nematodes, such as crop rotation with non-host crops or resistant cultivars (Molendijk and Sikora, 2021). Crop rotation to non-host crops suppresses *M. enterolobii* populations because it cannot reproduce without a suitable host (Niere and Karuri, 2018). Nematode populations can be reduced by rotating hosts for at least a year (McSorley, 2011). As a result, crops should rotate to non-hosts for at least three years (Seid et al., 2015). While crop rotation is impeded because of *M. enterolobii’s* vast variety of hosts (Groover, 2017). The rotation crops of garlic (*Allium sativum*), grapefruit (*Citrus paradise*), maize (*Zea mays*), peanut (*Arachis hypogaea*), sour orange (*C. aurantium*), and wheat can be used because they have been known to be poor hosts of *M. enterolobii* (Rodriguez et al., 2003). Additional cultural practices such as steaming, flooding, and soil solarization could be applied (Schwarz, 2019; Schwarz et al., 2020). A key prophylactic tactic is weed control, as many of them can act as *M. enterolobii*’s hosts (Bellé et al., 2019). Nematodes may spread rapidly through agricultural tools, water, and plant matter; thus, sterilization prevents the nematodes from spreading to unaffected fields (Philbrick et al., 2020). To promote the effective management of *M. enterolobii*, a more specific study on cultural control measures like soil amendments, crop rotational strategies, and tillage is required.

## Conclusion and perspectives

In this review, we particularly emphasized the advancements achieved by numerous researchers in biology, identification and control of *M. enterolobii*. The new outbreak of the extremely pathogenic and destructive nematode *M. enterolobii* threatens agriculture worldwide. Biological control with microbial antagonists (bacteria and fungi) has generated tremendous attention as a safe alternate and potential method of controlling *M. enterolobii* for ecological balance and safety. Extensive investments are required in fundamental research aimed at identifying species and understanding parasitism mechanisms, evolution, and genetic diversity at a deep level to control this emerging RKN. Therefore, it is more vital than ever to create accurate and reliable identifying genetic markers, specifically for proper identification and to restrict the emergence of this pathogenic RKN. Both traditional methods and modern technologies must be considered to maintain food security. Currently, researchers have also concentrated on finding alternative sources of genetic resistance against *M. enterolobii* because this species has the potential to reproduce on a variety of crops that have resistance genes against other nematodes species. The fresh insights on existing and forthcoming concerns, underpinned by only a better knowledge of the relationship between the host and *M. enterolobii*, may increase the potential for inventing new management strategies. Controlling such an economically destructive nematode in agricultural production systems must involve broad research alliances and bring multidisciplinary researchers studying *M. enterolobii*.

## Author contributions

AS, LJ and HW discussed and conceived ideas. AS gathered the literature and wrote the manuscript. HW and SY helped to revise the manuscript. All authors have read, edited, and approved it for publication.
